# Evaluation of Nursing Effect of Pelvic Floor Rehabilitation Training on Pelvic Organ Prolapse in Postpartum Pregnant Women under Ultrasound Imaging with Artificial Intelligence Algorithm

**DOI:** 10.1155/2022/1786994

**Published:** 2022-04-25

**Authors:** Ping Yin, Hongli Wang

**Affiliations:** ^1^Department of Gynecology, Hunan Maternity and Child Health Hospital, Changsha, 410008 Hunan, China; ^2^Settlement Center, Hunan Maternal and Child Health Hospital, Changsha, 410008 Hunan, China

## Abstract

This study was aimed at exploring the application value of ultrasound technology and rehabilitation training based on artificial intelligence algorithm in postpartum recovery of pelvic organ prolapse. Sixty patients diagnosed as mild and moderate pelvic organ prolapse by pelvic organ prolapse quantification evaluation were selected as the research objects. The patients were randomly divided into experimental group (30 cases) and control group (30 cases). The patients in the control group were given routine guidance and postpartum health education 42 days after delivery and given no pelvic floor rehabilitation training, waiting for natural recovery. 42 days after delivery, the patients in the experimental group received pelvic floor rehabilitation training based on the patients in the control group. All patients underwent ultrasonography, the convolution neural network (CNN) algorithm was used for image denoising and edge feature extraction, and the performance of the algorithm was evaluated by the Dice coefficient, positive predictive value, sensitivity, and Hausdorff distance. The thickness of levator ani muscle, anterior and posterior diameter of perineal hiatus, pelvic floor muscle strength, and imaging data were compared between the two groups. The results revealed that the thickness of levator ani muscle in the experimental group was significantly greater than that in the control group after one month and three months of treatment (0.633 ± 0.26 cm vs. 0.519 ± 0.234 cm, 0.7 ± 0.214 cm vs. 0.507 ± 0.168 cm, *P* < 0.05). After one month and three months of treatment, the anterior and posterior diameter of perineal fissure in the experimental group was obviously smaller than that in the control group (4.76 ± 0.513 cm vs. 5.002 ± 0.763 cm, 4.735 ± 0.614 cm vs. 4.987 ± 0.581 cm, *P* < 0.05). The pelvic floor muscle strength of the experimental group was remarkably higher than that of the control group after one month and three months of treatment (3.183 ± 1.47 vs. 2.41 ± 1.57, 3.365 ± 1.53 vs. 2.865 ± 1.69, *P* < 0.05). The ultrasonic image was clearer, the focus was more prominent, and the image quality was significantly improved after being processed by artificial intelligence algorithm. The Dice coefficient, positive predictive value, sensitivity, and Hausdorff distance of the proposed algorithm were better than those of the traditional algorithm. Thus, artificial intelligence algorithm had a good effect in ultrasonic image processing. Pelvic floor rehabilitation training had a good effect on postpartum nursing of patients with pelvic organ prolapse.

## 1. Introduction

Pelvic floor dysfunction (PFD) was a common gynecological disease. The main clinical manifestations were urinary loss, pelvic organ prolapse, fecal incontinence, and sexual dysfunction. The incidence rate was maintained at 20% to 40% [1]. Pregnancy and childbirth were the main causes of pelvic floor muscle injury. Data showed that about 40% of women suffered from pelvic floor muscles varying degrees of injury after birth, and the incidence rate increased [2, 3] with age. During pregnancy, the fetus continues to grow with the increase of the number of weeks of pregnancy, and the weight and amniotic fluid also increase. The increased uterine volume and weight leads to the position of the uterus from the anteversion area to the vertical axis perpendicular to the pelvic floor muscle. Moreover, perineal lateral incision or tear during delivery will directly damage the pelvic floor muscles, which can cause damage to the pelvic floor muscle tissue [4]. In recent years, with the increasing pressure of life, the population of late marriage and late childbearing in China has further increased. Meanwhile, the prevalence of pelvic floor dysfunction diseases has also further increased. Many studies indicated that the damage caused by pregnancy and delivery was reversible. This damage could be effectively repaired if timely and scientific care was taken after delivery [5, 6].

Pelvic floor rehabilitation training was one of the most effective methods for the treatment of pelvic floor dysfunction diseases. It mainly included pelvic floor muscle training (PFMT), pelvic floor rehabilitation assisted pelvic floor muscle exercise, pelvic floor biofeedback therapy, and electrical stimulation therapy [7]. Pelvic floor muscle exercise therapy is also known as Kegel training. Patients were allowed by Kegel training to consciously perform autonomous contraction on the pelvic floor muscles to achieve the purpose of increasing urine control [8]. Biofeedback therapy is a treatment method to help patients correctly identify the contraction signal of the pelvic floor muscle. The contraction signal of pelvic floor muscle was detected through the therapeutic probe placed in the vagina. Moreover, the contraction signal of the pelvic floor muscle was converted into visual information recognizable by the naked eye and prompted to the patient. The patients were helped receive the contraction signal and complete the contraction action [9]. Electrical stimulation (ES) referred to stimulating the pelvic floor muscle fibers through low current to cause regular contraction, so as to promote the recovery of pelvic floor muscle strength and the regeneration of the pudendal nerve [10]. At present, there is no conclusion on the best time of pelvic floor treatment. However, it was considered that after six months of delivery, women's lochia was basically drained, and the functions of the uterus, organs, and tissues were basically restored to normal. At this time, the pelvic floor could be effectively activated, the blood circulation of the pelvic floor muscles was accelerated, the repair and regeneration of perineal nerve structure and function were promoted, and the fibrosis of maternal pelvic floor tissue was reduced, so as the occurrence of pelvic floor dysfunction diseases was reduced, if the patients were given pelvic floor rehabilitation treatment [11].

There are many diagnostic methods for female pelvic floor dysfunction diseases, such as magnetic resonance imaging (MRI), CT, cystourethrography, and pelvic floor ultrasonography. The urodynamics of the lower urinary tract can be analyzed by cystourethrography. In addition, the anatomical structure of the female pelvic floor can also be shown by cystourethrography. However, cystourethrography has certain radioactivity, which limits its application. The pelvic floor tissue and structure can clearly be shown by MRI, but the changes of pelvic floor images in different states during scanning cannot be reflected by it, which has high requirements for patients and is expensive. With the rapid development of ultrasound technology, it was widely used in clinic with its unique advantages. Later, dynamic observation of three-dimensional anatomical structure of pelvic floor was provided with an effective method by the emergence of three-dimensional reconstruction technology [12]. Based on the above, ultrasound technology was more and more widely used in the clinical diagnosis of pelvic floor dysfunction diseases. However, the pressure on doctors to read films was increasing. In addition, the traditional diagnostic methods were deeply affected by doctors' subjective judgment and experience. It was easy to cause misdiagnosis and missed diagnosis. In recent years, computer technology continues to mature, and some image processing technologies are becoming more and more perfect and mature. These technologies were applied in medical image processing. Artificial intelligence algorithm was one of the most widely used and concerned technologies in the field of medical images. It showed excellent performance in medical image feature extraction, lesion segmentation, noise reduction, and edge detection [13]. At present, there are few studies on the application of this technology in ultrasonic image processing of pelvic floor dysfunction diseases. Artificial intelligence algorithm was used to process and optimize the ultrasound images of patients with pelvic floor dysfunction diseases. On this basis, the effect of pelvic floor rehabilitation training on postpartum pelvic floor tissue structure and function recovery was explored. It was expected to provide reference and basis for the diagnosis and treatment of clinically related diseases.

## 2. Research Materials and Methods

### 2.1. Research Object

Sixty patients in hospital from March 2019 to September 2020 were selected as the research object. The average age of the patients was 34.6 ± 11.5 years. All selected patients were diagnosed as mild and moderate pelvic organ prolapse by pelvic organ prolapse quantification (POP-Q) evaluation. The patient's medical history, gynecological examination, pop evaluation, B-ultrasound data, and pelvic prolapse were collected. The patients were randomly divided into experimental group (30 cases) and control group (30 cases). Inclusion criteria are as follows: patients aged 25 to 65 years, with mild and moderate pelvic prolapse, namely, POP-Q score of grades I ~ II. Patients were able to complete regular follow-up. The informed consent was obtained from patients and this study had been approved by the medical ethics committee of hospital. Exclusion criteria are as follows: patients with acute inflammation of the urinary and reproductive tract, pelvic tumor, history of pelvic surgery, sciatica, and other neurological diseases.

### 2.2. Ultrasonic Examination Method

The color Doppler ultrasound diagnostic instrument and variable frequency vaginal probe were used. Before the examination, the patient was instructed to empty the bladder without residual urine. The bladder lithotomy position was taken, and the sagittal section was examined with the vaginal probe. The probe was externally plied with a disposable condom, the surface was coated with neutral coupling agent, the labia majora was separated, the upper edge was close to the lower edge of the pubic symphysis, and the junction of the pubic symphysis, urethra, anal canal, and rectum could be clearly displayed. Three-dimensional imaging was performed to clearly show the minimum plane of the pelvic genital hiatus, and the urethra, vagina, and anus could be seen at the same time after imaging.

### 2.3. Image Optimization

All the images obtained were optimized by convolution neural network algorithm (CNN). CNN can directly take the original medical image as the initial input data of the processing process. By learning the weight information features, CNN can simplify the feature extraction part of the steps of the traditional recognition algorithm. It was a popular and widely used algorithm at present. It mainly included two parts: denoising and image feature extraction. The specific details were as follows.

Denoising: for an array with *f*(x, y) as *g*(x, y). After processing, the image was *g*(x, y), and its gray level was determined by the average of the gray levels of several pixels in the (x, y) field. The representation of the processed image was as follows.

(1) $$\begin{array}{c} g\left(x,y\right)=\frac{1}{M}\underset{\left(i,j\right)\in s}{\sum }f\left(i,j\right). \end{array}$$

*x*, *y* = 0, 1, 2 ⋯ , N − 1 and *S* were the domain set centered on point (x, y), and M is the total number of coordinate points in point *S*.

For multiple images, if the original image was *f*(x, y) and the image noise was *n*(x, y), the noisy image *g*(x, y) was as follows.

(2) $$\begin{array}{c} g\left(x,y\right)=f\left(x,y\right)+n\left(x,y\right). \end{array}$$

If the noise was uncorrelated and the mean value was zero, then equation (3) was obtained.

(3) $$\begin{array}{c} f\left(\text{x},\text{y}\right)=\text{E}\left[g\left(\text{x},\text{y}\right)\right], \end{array}$$

where E[*g*(x, y)] was the expected value of *g*(x, y). M noisy images were averaged, then equations (4) and (5) were obtained.

(4) $$\begin{array}{c} f\left(\text{x},\text{y}\right)=\text{E}\left[g\left(\text{x},\text{y}\right)\right]\sim \bar{g}\left(\text{x},\text{y}\right)=\frac{1}{M}\overset{M}{\underset{i=1}{\sum }}g_{i}\left(\text{x},\text{y}\right), \end{array}$$

(5) $$\begin{array}{c} {\delta^{2}}_{\bar{g}\left(\text{x},\text{y}\right)}=\frac{1}{M}{\delta^{2}}_{n\left(\text{x},\text{y}\right)}. \end{array}$$

In the above equations, ${\delta^{2}}_{\bar{g}\left(\text{x},\text{y}\right)}$ and *δ*^2^_*n*(x, y)_ were the variances of $\bar{g}$ and *n* at point (x, y).

Edge detection and equation (6) were obtained.

(6) $$\begin{array}{c} \psi^{2}\left(\text{x}\right)=\frac{d^{2}\theta \left(\text{x}\right)}{{dx}^{2}}. \end{array}$$

Definition of equation (7) was as follows.

(7) $$\begin{array}{c} w^{1}f\left(s,x\right)=f*\psi_{s}^{1}\left(x\right)w^{2}f\left(s,x\right)=f*\psi_{s}^{2}\left(x\right), \end{array}$$

(8) $$\begin{array}{c} w^{1}f\left(s,x\right)=f*\left(s\frac{d\theta_{s}}{dx}\right)\left(x\right)=s\frac{d}{dx}\left(f*\theta_{s}\right)\left(x\right), \end{array}$$

(9) $$\begin{array}{c} w^{2}f\left(s,x\right)=f*\left(s^{2}\frac{d^{2}\theta_{s}}{{dx}^{2}}\right)\left(x\right)=s^{2}\frac{d^{2}}{{dx}^{2}}\left(f*\theta_{s}\right)\left(x\right). \end{array}$$

The membrane value of point W_2^*j*^_^1,d^*f*(n, m), W_2^*j*^_^2,d^*f*(n, m) and point (n, m) of discrete dyadic wavelet transform could be obtained in equation (10).

(10) $$\begin{array}{c} M_{2^{j}}^{d}f\left(n,m\right)=\sqrt{{\left|W_{2^{j}}^{1,d}f\left(n,m\right)\right|}^{2}+{\left|W_{2^{j}}^{2,d}f\left(n,m\right)\right|}^{2}}. \end{array}$$

The phase angle was obtained as follows.

(11) $$\begin{array}{c} A_{2^{j}}^{d}f\left(n,m\right)=\arg\tan\left(\frac{W_{2^{j}}^{2,d}f\left(n,m\right)}{W_{2^{j}}^{1,d}f\left(n,m\right)}\right). \end{array}$$

Four indexes were used to evaluate the performance of the algorithm: the Dice coefficient, positive predictive value, sensitivity, and Hausdorff distance.

### 2.4. Training Methods

The control group is as follows: the patients in the control group were given routine guidance and postpartum health education 42 days after delivery: the patients were told the impact of delivery on pelvic floor function and postpartum pelvic floor health care knowledge. The pregnant women were instructed to maintain good health habits and master correct urination methods. No pelvic floor rehabilitation training was carried out to the patients in the control group, waiting for natural recovery.

The experimental group is as follows: 42 days after delivery, the patients in the experimental group were given pelvic floor rehabilitation training: electrical stimulation, biofeedback, and PFMT based on the patients in the control group.

Electrical stimulation and biofeedback are as follows: the pregnant women emptied their urine first and stayed in the semirecumbent position, relaxed naturally, and slightly separated their thighs (the pregnant women were instructed to prohibit abdominal pressure during vaginal muscle contraction). The EMG pelvic floor muscle treatment head was placed into the vagina, and the electrical stimulation current intensity gradually increased from 0 mA. The maximum current intensity of treatment stimulation shall be subject to the maternal feeling of stimulation but no pain. The muscle strength was adjusted at the contraction site according to the biofeedback signal. Electrical stimulation and biofeedback should be conducted 30 min/time, 2 times/week, and 10 times/course of treatment.

PFMT is as follows: the pregnant women were instructed to contract continuously and alternately and to relax the pelvic floor muscles and levator ani muscles. The levator ani exercises lasted for about 7 s and relaxed for about 7 s. Each time was 10 min to 15 min, and 3 times to 8 times a day, lasting for 8 weeks or more.

### 2.5. Statistical Analysis

All data analysis was completed by the SPSSl9.0 statistical software. The measurement data was represented by $\bar{x}+s$ test, independent sample *t* test, and the comparison between groups is completed by *x*^2^ test. The nonparametric rank sum Mann–Whitney *U* test of independent samples was used for the above samples, and the difference was statistically significant (*P* < 0.05).

## 3. Results

### 3.1. General Information of Patients

The general data of the two groups are illustrated in Table 1. It was revealed that the average age of the patients in the experimental group was years, the weight was kg, and the average height was m. The average age of the control group was years, the weight was kg, and the average height was m. Therefore, there was no significant difference in height, weight, and age between the two groups. Table 1 also presents that there was no significant difference between the two groups in fertility, mode of delivery, diagnosis, and other data. Therefore, the two groups of patients were comparable.

### 3.2. Ultrasonic Image Display of Typical Cases

The ultrasound images of the two groups of typical cases in each time period are shown in Figures 1 and 2. It was found that the recovery of the experimental group was better than that of the control group at the same time. After the two groups of images were processed by artificial intelligence algorithm, the images were clearer, the lesions were more prominent, and the image quality was significantly improved.

### 3.3. Evaluation Index of Algorithm Processing Performance

The performance evaluation results of the traditional algorithm and the proposed algorithm are shown in Figure 3. The Dice coefficient, positive predictive value, sensitivity, and Hausdorff distance of the proposed algorithm were 0.81, 0.98, 0.93, and 1.2, respectively; the Dice coefficient, positive predictive value, sensitivity, and Hausdorff distance of the traditional algorithm were 0.66, 0.71, 0.62, and 3.3, respectively. Compared with the two algorithms, the performance of CNN algorithm in ultrasonic image segmentation was significantly better than that of the traditional algorithm, *P* < 0.05.

### 3.4. Comparison of Ultrasonic Indexes between the Two Groups before and after Treatment

The comparison results of two-dimensional ultrasound and three-dimensional ultrasound indexes before and after treatment in the experimental group are shown in Figures 4 and 5. According to the analysis of Figure 4, the distance between the bladder bottom and the posterior line of the pubic symphysis in the experimental group was prolonged. According to the analysis of Figure 5, it was shown in three-dimensional ultrasound that the puborectalis muscle was thicker and the anterior and posterior diameter of perineal hiatus was significantly shorter than that before treatment.

The comparison results of two-dimensional ultrasound and three-dimensional ultrasound indexes before and after treatment in the control group are shown in Figures 6 and 7. According to the analysis of Figure 6, it was shown in two-dimensional ultrasound that the distance between the anal junction and the posterior line of the pubic symphysis increased. According to the analysis of Figure 7, the puborectal muscle was thickened and the anterior and posterior diameter of perineal hiatus was shortened under the contraction of levator ani muscle.

### 3.5. Comparison of Levator Ani Muscle Thickness before and after Treatment

The comparison results of levator ani muscle thickness between the experimental group and the control group before and after treatment are shown in Figure 8. According to the analysis of Figure 8, there was significant difference in the thickness of levator ani muscle between the experimental group and the control group after treatment for one month and three months, *P* < 0.05.

### 3.6. Comparison of Perineal Fissure Diameter before and after Treatment

The comparison results of the anterior and posterior diameter of perineal holes between the experimental group and the control group before and after treatment are shown in Figure 9. According to the analysis of Figure 9, there was significant difference in the diameter of perineal fissure between the experimental group and the control group after treatment for one month and three months, *P* < 0.05.

### 3.7. Comparison of Pelvic Floor Muscle Strength between the Two Groups

The comparison results of pelvic floor muscle strength between the two groups before and after treatment are shown in Figure 10. According to the analysis of Figure 10, there was significant difference in pelvic floor muscle strength between the experimental group and the control group after treatment for one month and three months, *P* < 0.05.

## 4. Discussion

PFD refers to a series of clinical symptoms caused by weak pelvic floor function due to various reasons, mainly including urinary incontinence, pelvic organ prolapse, sexual dysfunction, and fecal incontinence. At present, the pathogenesis is not clear. Clinically, its pathogenesis is generally divided into four stages, namely, susceptibility factors, promotion conditions, progression, and dysfunction. Many studies showed that pregnancy and vaginal delivery were one of the essential and main causes of PFD [14]. Epidemiological studies showed that 20% ~40 parturients had urinary incontinence within four months postpartum, while the probability of urinary incontinence within twelve months postpartum was 30.5%. In addition, the incidence of sexual dysfunction in primipara was 70.6% [15]. In summary, it is suggested that pregnancy and delivery are the most important and key factors leading to pelvic floor dysfunction. Although the incidence rate of post pelvic floor dysfunction diseases is very high, it is fortunate that clinical studies show that most of the pelvic floor dysfunction diseases are reversible and can be repaired by some rehabilitation treatments.

The treatment of pelvic floor dysfunction can be divided into two categories: surgical treatment and nonsurgical treatment. Surgical treatment has many disadvantages, such as large trauma, high cost, postoperative complications, and high recurrence rate. Therefore, pelvic floor rehabilitation has become a research hotspot in recent years. Some scholars pointed out that pelvic floor muscle exercise was performed at 8 weeks postpartum, and the incidence of urinary incontinence and pelvic floor prolapse in the experimental group was significantly lower than that in the control group at 16 weeks and one-year postpartum. Moreover, the study also pointed out that attention should be paid to the frequency and intensity of exercise [16]. Pelvic floor rehabilitation treatment mainly includes pelvic floor muscle exercise, biofeedback, and electrical stimulation. At present, there is no unified theory on which of the three treatments is better. In addition, clinical studies tend to combine the three methods for comprehensive treatment of pelvic floor dysfunction [17].

The position of various organs in the pelvic floor can be clearly displayed by pelvic floor ultrasound. The organ prolapse of each chamber can be visually observed and quantitatively analyzed by pelvic floor ultrasound, which provides detailed pelvic floor morphological and functional information for clinical practice, and is beneficial to identify the type of prolapse. Based on the above advantages, ultrasound is widely used in the diagnosis of pelvic floor diseases [18, 19]. However, with the deepening of people's understanding of diseases, people's requirements for the quality of ultrasonic images are also improving. In recent years, with the continuous progress and development of computer and Internet technology, some image processing technologies were also improved and developed, and they were penetrated into many fields [20]. Medical image processing technology was one of the more important and popular research fields [21]. Artificial intelligence algorithm was one of the most concerned and promising algorithms. It made some achievements and progress in the field of medical image processing, such as the proposal of some computer-aided diagnosis systems [22]. However, the current research on artificial intelligence algorithms in the medical field mostly focused on the segmentation of tumor or hemorrhagic disease lesions, and there was almost no application on pelvic floor injury diseases [23, 24].

Patients with pelvic organ prolapse were studied, all patients underwent ultrasonography, and all image maps were processed by CNN. On this basis, the effect of pelvic floor rehabilitation training on postpartum recovery of parturients with pelvic floor organ prolapse was explored. It was found that the parturients in the experimental group who had received rehabilitation training were superior to the parturients in the control group who had not received rehabilitation treatment in terms of pelvic floor muscle strength, levator ani muscle thickness, anteroposterior diameter of perineal hiatus, and ultrasound findings. The ultrasound images processed by artificial intelligence algorithm were clearer than the untreated images, with more prominent lesions and significantly improved image quality, providing a reference and basis for postpartum pelvic floor rehabilitation training and parturients' pelvic organ prolapse nursing in clinical practice. Therefore, appropriate pelvic floor training in the postpartum period is effective for reducing the occurrence of postpartum pelvic prolapse and helping pelvic floor muscle recovery, which is consistent with the results of previous studies.

## 5. Conclusion

Patients with pelvic organ prolapse were studied. All patients underwent ultrasonography, and all images were processed by artificial intelligence algorithm. On this basis, the effect of pelvic floor rehabilitation training on postpartum recovery of pregnant women with pelvic floor organ prolapse was explored. It was found that compared with the pregnant women undergoing rehabilitation training, the experimental group was better than the control group in pelvic floor muscle strength, levator ani muscle thickness, perineal fissure anterior and posterior diameter, and ultrasonic performance. Compared with the untreated images, the ultrasound images processed by artificial intelligence algorithm are clearer, the lesions are more prominent, and the image quality is significantly improved. In conclusion, pelvic floor rehabilitation training has a good effect on postpartum recovery of pregnant women with pelvic organ prolapse, and artificial intelligence algorithm has a good effect on ultrasonic image processing. Due to the limited samples and space, it is not comprehensive and in-depth. In the future, more samples will be added to further explore the problem comprehensively and in-depth.

## Figures and Tables

**Figure 1:** Ultrasonic images of experimental group at each time period.

**Figure 2:** Ultrasound images of the control group at each time period.

**Figure 3:** Quantitative evaluation results of image processing performance. ^∗^Compared with CNN, *P* < 0.05.

**Figure 4:** Comparison of two-dimensional ultrasound indexes of patients in the experimental group before and after treatment. (a) the distance from bladder bottom to posterior line of the pubic symphysis; (b) the distance from the cervix to pubic symphysis; (c) the distance between the connecting part of the anal canal and the posterior connecting line of the pubic symphysis. ^∗^Compared with before treatment, *P* < 0.05.

**Figure 5:** Comparison of three-dimensional ultrasound indexes of patients in the experimental group before and after treatment. (a) Anteroposterior diameter of perineal foramen; (b) area; (c) puborectal muscle thickness. ^∗^Compared with before treatment, *P* < 0.05.

**Figure 6:** Comparison of two-dimensional ultrasound indexes in the control group before and after treatment. (a) Distance from bladder bottom to posterior line of pubic symphysis; (b) the distance from the cervix to the pubic symphysis; (c) the distance between the connecting part of the anal canal and the posterior connecting line of the pubic symphysis. ^∗^Compared with before treatment, *P* < 0.05.

**Figure 7:** Comparison of three-dimensional ultrasound indexes in the control group before and after treatment. (a) Anteroposterior diameter of perineal foramen; (b) area; (c) puborectal muscle thickness. ^∗^ Compared with before treatment, *P* < 0.05.

**Figure 8:** Comparison of levator ani muscle thickness between the two groups before and after treatment. ^∗^Compared with the experimental group, *P* < 0.05.

**Figure 9:** Comparison of anterior and posterior diameter of perineal hiatus between the two groups before and after treatment. ^∗^Compared with the experimental group, *P* < 0.05.

**Figure 10:** Comparison of pelvic floor muscle strength between the two groups before and after treatment. ^∗^Compared with the experimental group, *P* < 0.05.

**Table 1:** General information of patients.

Items		Experimental group	Control group	*P*
Age (years)		38.55 ± 5.38	39.9 ± 6.37	0.63
Weight (kg)		55.70 ± 10.21	56.9 ± 7.78	0.77
Height (m)		1.62 ± 0.02	1.59 ± 0.03	1.2
Fertility	1	13	14	1.1
	≥2	17	16	3.2
Mode of delivery	Cesarean section	18	16	0.8
	Forceps	12	14	0.09
Diagnosis	I	16	15	2.2
	II	14	15	1.1

## Data Availability

The data used to support the findings of this study are available from the corresponding author upon request.
